This article has been retracted.

# MiR-143-3p functions as a tumor suppressor by regulating cell proliferation, invasion and epithelial–mesenchymal transition by targeting QKI-5 in esophageal squamous cell carcinoma

**DOI:** 10.1186/s12943-016-0533-3

**Published:** 2016-06-29

**Authors:** Zhenyue He, Jun Yi, Xiaolong Liu, Jing Chen, Siqi Han, Li Jin, Longbang Chen, Haizhu Song

**Affiliations:** Department of Medical Oncology, Jinling Hospital, Medical School of Nanjing University, 305 Zhongshan East Road, Nanjing, Jiangsu 210002 People’s Republic of China; Department of Cardiothoracic Surgery, Jinling Hospital, Medical School of Nanjing University, 305 Zhongshan East Road, Nanjing, Jiangsu 210002 People’s Republic of China

**Keywords:** MiR-143-3p, Esophageal squamous cell carcinoma, QKI-5, Proliferation, Invasion

## Abstract

**Background:**

Dysregulation of microRNAs (miRNAs) have been demonstrated to contribute to carcinogenesis. MiR-143-3p has been identified to function as a tumor suppressor in several tumors, but the role of miR-143-3p in esophageal squamous cell carcinoma (ESCC) has not been intensively investigated. Our aim was to evaluate the potential role of miR-143-3p in the progression of ESCC.

**Methods:**

The expression levels of miR-143-3p and QKI-5 protein were measured in 80 resected ESCC tumor specimens and the clinicopathological significance of these levels determined. We also investigated the role of miR-143-3p in the regulation of QKI-5 expression in ESCC cell lines both in vivo and in vitro.

**Results:**

MiR-143-3p levels were decreased in ESCC clinical samples and low expression of miR-143-3p was significantly associated with poor prognosis in ESCC patients. Ectopic expression of miR-143-3p suppressed proliferation and induced apoptosis in ESCC cells both in vivo and in vitro. Ectopic expression of miR-143-3p also reduced the metastatic potential of cells by selectively regulating epithelial–mesenchymal transition regulatory proteins. Furthermore, QKI-5 isoform was upregulated in ESCC tissues and was a direct target of miR-143-3p. Lastly, re-introduction of QKI-5 expression abrogated the inhibitory effects of miR-143-3p on ESCC cell proliferation and motility.

**Conclusions:**

Our results demonstrate that miR-143-3p acts as a tumor-suppressor by targeting QKI-5 in ESCC, suggesting that miR-143-3p is a potential therapy for the treatment of ESCC.

**Electronic supplementary material:**

The online version of this article (doi:10.1186/s12943-016-0533-3) contains supplementary material, which is available to authorized users.

## Background

Esophageal cancer (EC) is the eighth-most common cancer with a highly aggressive potency, and the sixth leading cause of cancer-related mortality worldwide [1]. The two main types of EC are esophageal adenocarcinoma (EA) and esophageal squamous cell carcinoma (ESCC), and each disease possesses distinct histopathological features and clinical behaviors. ESCC is the most frequent subtype of EC, with EA less common in China. Epidemiological study indicates that the incidence and histological subtypes of EC are associated with environmental, genetic and epigenetic factors [2]. No typical symptoms suggestive of ESCC exist until disease is advanced, conferring difficulty upon early diagnosis of ESCC. Moreover, the limited medical and surgical treatment options for patients diagnosed at a later stage underpin a poor prognosis with a 5-year overall survival rate of 15–25 % [3]. Exploration of the molecular mechanisms that promote ESCC development and progression could improve the diagnosis, therapy, and prevention of this disease.

MicroRNAs (miRNAs) are endogenous non-coding RNAs of 18–22 nucleotides in length that regulate gene expression by complementary binding to the 3’-untranslated regions (3’-UTR) of specific mRNA targets [4, 5]. Accumulating evidence suggests that dysregulated miRNAs can function either as oncogenes or tumor suppressor genes to affect the initiation and progression of tumors, including ESCC [6–9]. A previous study identified miR-21 upregulation in ESCC cell lines and tissues, with increased miR-21 promoting cell proliferation and invasion by targeting PTEN and PDCD4 [10]. Another study has revealed that miR-145, miR-133a and miR-133b suppressed tumor proliferation by regulating the oncogenic actin-binding protein, FSCN1 [11].

The QKI protein belongs to the signal transduction and activation of RNA (STAR) protein family and is a key post-transcriptional regulator. *QKI* expresses three major alternatively spliced mRNAs: QKI-5, QKI-6 and QKI-7. QKI-5 is the only nuclear isoform and shuttles between the nucleus and cytoplasm [12], whereas QKI-6 is distributed throughout the cell and QKI-7 is cytoplasmic [13]. These QKI proteins selectively interact with the QKI response element and function in various aspects of RNA processing [14, 15]. Aberrant expression of QKI-5 is associated with the development and progression of human cancers. For example, QKI-5 functions as a tumor suppressor gene in prostate cancer [16] and colon cancer [17]. However, the potential role for QKI-5 in ESCC proliferation and metastasis has not been described.

Our present study demonstrates that miR-143-3p, a miRNA species that is downregulated in ESCC tissues and cell lines, inhibits the development and metastasis of ESCC cells both in vivo and in vitro. Specifically, our study reports for the first time that QKI-5 is a direct target of miR-143-3p in ESCC. MiR-143-3p-dependent downregulation of QKI-5 inhibited cell proliferation, migration, and invasion of ESCC cells. These findings indicate that the miR-143-3p/QKI-5 axis is an important regulator of the development and progression of ESCC and provides a candidate target for ESCC treatment.

## Methods

### Cell culture and tissue samples

The human normal esophageal epithelial cell line HEEC and human ESCC cell lines (Kyse30, Kyse70, Eca109, and Ec9706) were purchased from the Cell Bank of Shanghai Institute of Cell Biology (Chinese Academy of Medical Sciences, Shanghai, China). HEEC, Kyse30, Kyse70, and Eca109 cells were expanded in RPMI-1640 medium (Gibco, USA) supplemented with 10 % fetal bovine serum (FBS, Gibco, USA) and 1 % penicillin/streptomycin (Invitrogen, Shanghai, China). Ec9706 cells were grown in Dulbecco’s modified eagle’s medium (DMEM, Gibco, USA) supplemented with 10 % FBS and 1 % penicillin/streptomycin. Cells were all cultured at 37 °C in a 5 % CO_2_ -humidified incubator.

Pairs of primary ESCC and adjacent normal tissue specimens (*n* = 80) were obtained from the Cardiothoracic Surgery Department of Jinling Hospital (Jiangsu, China). None of the patients with ESCC had received radiotherapy or chemotherapy before surgery. The research protocol was reviewed and approved by the Ethical Committee and Institutional Review Board of the Jinling Hospital, and written informed consent was obtained from each patient included in the study.

### MiRCURY LNA array analysis

Total RNA was extracted from five pairs of ESCC tumor and adjacent normal tissues using the mirVana miRNA isolation kit (Ambion, USA). Microarray chip analysis was performed and analyzed by Exiqon (Vedbaek, Denmark). The fold-change was calculated by comparing the expression level of miRNAs in the ESCC tumor pool and with that of the normal tissue pool using a log_2_ format.

### miRNA target prediction

Five established miRNA-target prediction programs (TargetScan, miRanda, PicTar, MirTarget2, and PITA) were employed to predict miRNA targets, with genes predicted by all five independent tools considered. The selected genes of each individual miRNA were subjected to GO and pathway analysis.

### Plasmid and cell transfection

We selected Kyse30, Kyse70, and Eca109 cells for further functional research. Plasmids encoding miR-143-3p, anti-miR-143-3p and their corresponding controls (miR-NC and anti-miR-NC) were purchased from ABM (ABM, Canada). For the reduction and induction of QKI-5 expression, GFP-tagged of human pLenti QKI-5, pLenti siQKI-5 and matched controls (pLenti-Blank and Scrambled siRNA) plasmids were also purchased from ABM (ABM, Canada). Cells were transfected with plasmids using DNAfectin Plus (ABM, Canada) according to the manufacturer’s protocol. Stably-transfected cells were selected for 14 days in the presence of 2 μg/mL puromycin (Sigma, USA).

### Western blot analysis

Cells and tissues were lysed with ice-cold RIPA buffer supplement with Phenylmethanesulfonyl Fluoride (PMSF) and cocktail. Total protein concentrations were measured using the KeyGEN BCA Protein Quantitation Assay (KeyGEN, China). Cell lysates were subjected to sodium dodecyl sulfate-polyacrylamide gel electrophoresis and transferred onto polyvinylidene fluoride membranes. Membranes were incubated with the following primary antibodies overnight at 4 °C: rabbit anti-human QKI antibody (Bethyl, USA), epithelial-mesenchymal transition antibody (Cell Signaling, USA), and mouse anti-human GAPDH antibody (Cell Signaling, USA). Membranes were then incubated with horseradish peroxidase-conjugated goat anti-rabbit or goat anti-mouse antibody for 1 h at 37 °C. Immunoreactive bands were visualized using an enhanced ECL system (Thermo Scientific, USA) and the blots were exposed to Kodak X-ray film. Quantification of western blots was obtained by multiplying the area and intensity of each band using Image J software.

### Immunohistochemistry

Formalin-fixed paraffin-embedded tissue specimens were sectioned into 3–4 μm sections for immunohistochemistry. Sections were then treated with xylene, and hydrated through a series of decreasing concentrations of ethanol to water. For antigen retrieval, slides were incubated with citrate buffer solution (Maixin Bio, China) at 100 °C for 1 min. Slides were then immersed in 100 μl 3 % hydrogen peroxide for 10 min at room temperature, and the tissue sections incubated with primary antibody at 4 °C overnight. Subsequently, the sections were incubated with secondary antibody for 60 min at 37 °C. Last, diaminobenzidine was used as the colorizing reagent, and hematoxylin was used to counter stain nuclei.

Stained sections were scored by three pathologists independently and interobserver agreement reached. Each section was scored according to the intensity and percentage of positive cells. Staining intensity was scored as follows: 0 (negative), 1 (weakly positive), 2 (moderately positive), and 3 (strongly positive). The percentage of positive cells was also graded according to four categories, 1 point for 0–25 % positive cells; 2 for 26–50 % positive cells; 3 for 51–75 % positive cells; and 4 for more than 75 % positive cells. Overall scores ≤ 3 were defined as negative, and scores > 3 were defined as positive.

### RNA extraction, reverse transcription, and real-time quantitative RT-PCR

Total RNA was extracted from surgical tissue specimens and cell lines using TRIzol reagent (Takara, Japan) according to the manufacturer’s instructions. For miRNA reverse transcription, cDNA was synthesized using the miRNA cDNA Synthesis Kit (ABM, Canada). For mRNA reverse transcription, cDNA was synthesized using 5× All-In-One RT MasterMix (ABM, Canada). Real time quantitative RT-PCR was performed using EvaGreen miRNA qPCR Mastermix-ROX and EvaGreen 2× qPCR MasterMix-ROX (ABM, Canada) according to the manufacturer’s instructions. Relative quantification was achieved by normalization to the amount of *U6* (abbreviation of RNU6B) or *GAPDH* mRNA. All reactions were performed in triplicate. The primers for miR-143-3p and U6 were purchased from ABM. The primers for GAPDH were 5’-GCACCGTCAAGGCTGAGAAC-3’ and 5’-TGGTGAAGACGCCAGTGGA-3’. The primers for QKI-5, QKI-6, and QKI-7 have been described previously [18]. Relative gene expression levels were calculated by the ΔΔCt method.

### Cell proliferation assay

Cell proliferation was analyzed using the 3-(4, 5-dimethylthiazol-2-yl)-2, 5-diphenyltetrazolium bromide (MTT) assay. In total, 5 × 10^3^ transfected cells were seeded into each well of a 96-well plate and cultured for 1–3 days, followed by addition of MTT solution to the cells for 4 h. After removing the medium, the remaining MTT formazan crystals were solubilized in DMSO and absorbance was measured using a microplate reader at 490 nm.

### Colony formation assay

Transfected cells were seeded into six-well plates in triplicate (500 cells/well). Cells were allowed to grow for 10–14 days. To visualize colonies, cells were fixed with methanol and stained with 0.1 % crystal violet. Colonies with ≥ 50 cells were manually counted under a dissection microscope.

### Apoptosis assay

Cell apoptosis analysis was performed using an Annexin V-FITC/PI Apoptosis Detection Kit (Oncogene Research Products). Approximately 48 h after transfection, cells were digested with trypsin, washed twice with PBS, and then resuspended in the binding buffer. Annexin V-FITC and propidium iodide (PI) were then added. Finally, apoptosis was assessed by flow cytometry. The degree of apoptosis in tissue was also quantified using a TUNEL kit (Roche, Shanghai, China) according to the manufacturer’s instructions.

### In vitro migration and invasion assays

The wound healing assay was performed to assess cell migration ability. 5 × 10^5^ transfected cells were seeded into six-well plates. After serum starvation in serum-free medium for 24 h, an artificial wound was created on the confluent cell monolayer using a standard 200 μL plastic pipette tip. Cells migrated into the scratch area as single cells from the confluent sides, and the width of the scratch gap was viewed under an inverted microscope and photographed at 0 h and 48 h. Three replicates of each condition were used.

For the Transwell migration assay, the above transfected cells were plated to the upper chambers of 8-μm pore size Transwell plates (Corning, MA, USA). For the Matrigel-coated Transwell invasion assay, Matrigel and transfected cells were plated to the upper chambers of Transwell plates. All experiments were performed at least three times in triplicate. Approximately 24 h after seeding, cells that appeared on the undersurface of the filter were fixed with methanol, stained with 0.1 % crystal violet and counted under a microscope.

### Luciferase reporter assay

The luciferase reporter assays was conducted according to the manufacturer’s instructions (Promega, USA). Each sample was measured in triplicate, and the experiment was repeated at least three times. The transfection efficiency was measured by cotransfection with a *Renilla* luciferase expression plasmid pRL-SV40 (Promega, USA) and the luciferase activity was measured using the Dual-Luciferase Reporter Assay System (Promega, USA).

### Mice xenograft models and immunohistochemistry analysis

This study and all experimental protocols were approved by the authors’ institutional review board. Age-matched BALB/C nude mice were obtained from the Department of Comparative Medicine in Jinling Hospital. Approximately 5 × 10^6^ Kyse70 cells were suspended in 100 μL PBS and inoculated subcutaneously into the right side of the posterior flank of the mice. Beginning day 6 after injection, tumor diameters were measured every other day. After 18 days, all mice were killed, and necropsies were performed. Tumor volume was calculated using the equation: V = A × B^2^/2 (mm^3^), where A is the largest diameter and B is the perpendicular diameter. The primary tumors were excised and analyzed by immunohistochemistry and TUNEL staining.

### Statistical analysis

The categorical variables of the 80 clinical specimens examined were compared using the chi-square test. Survival analysis using the Kaplan-Meier method was performed using the log-rank test. The relationship between two variables and numerical values obtained by real-time quantitative RT-PCR were analyzed using Student’s *t*-tests. Multiple group comparisons were analyzed with one-way ANOVA. Statistical significance was defined as *P* <0.05. All statistical analyses were performed using SPSS18.0 software (SPSS Inc., USA).

## Results

### MiR-143-3p is frequently downregulated in ESCC cell lines and tissues

The roles of miRNA in ESCC were investigated by using miRCURY LNA array analysis to compare miRNA expression profiles between ESCC tumors and matched adjacent normal tissue specimens from five primary ESCC cases treated by the Cardiothoracic Surgery Department of Jinling Hospital. After global normalization of the raw data, 28 differentially expressed miRNAs were identified in ESCC tumor tissues compared with their normal tissues when using a 50-fold change cut-off point (Table 1). These included 21 highly-expressed miRNAs and seven lowly-expressed miRNAs.

**Table 1:** Differentiated dysregulation of miRNAs in ESCC

miRNA	Fold change	
hsa-miR-375	379.73	down
hsa-miR-143-3p	155.66	down
hsa-miR-133b	137.29	down
hsa-miR-143-5p	123.49	down
hsa-miR-29c-3p	121.19	down
hsa-miR-4649-3p	97.06	down
hsa-miR-100-5p	51.45	down
hsa-miR-630	182.20	up
hsa-miR-4419a	150.93	up
hsa-miR-4667-5p	120.98	up
hsa-miR-6131	110.54	up
hsa-miR-1183	106.78	up
hsa-miR-5703	105.74	up
hsa-miR-4306	105.03	up
hsa-miR-3692-5p	98.86	up
hsa-miR-6717-5p	96.40	up
hsa-miR-4476	92.87	up
hsa-miR-4665-5p	91.85	up
hsa-miR-3917	85.52	up
hsa-miR-3682-3p	85.04	up
hsa-miR-4419b	84.27	up
hsa-miR-3620-5p	83.90	up
hsa-miR-3194-5p	83.40	up
hsa-miR-4732-5p	81.94	up
hsa-miR-345-3p	81.64	up
hsa-miR-4496	81.26	up
hsa-miR-4738-3p	75.93	up
hsa-miR-3138	74.75	up

We further validated the microarray results by detecting the expression levels of the three most downregulated miRNAs (miR-143-3p, miR-133b, miR-143-5p) in the HEEC cell line and four ESCC cell lines. Figure 1a reveals that miR-143-3p exhibited the largest absolute fold-change in the expression in ESCC cell lines. We further measured the expression of miR-143-3p in 80 pairs of primary ESCC tissue specimens. Consistent with the above results, miR-143-3p was downregulated in primary tumor tissue specimens compared with the normal controls (Fig. 1b).

**Fig. 1:** MiR-143-3p is downregulated in ESCC cell lines and tumor tissue, and is associated with poor prognosis. **a** Real time RT-PCR analysis of three most differentially downregulated miRNAs expression in four human ESCC cell lines and the normal esophageal epithelial cell line (HEEC). **b** Real time RT-PCR analysis of miR-143-3p expression in 80 human ESCC tissue samples and their matched normal tissues. Expression levels are shown in log_2_ scale. **c** Correlation between miR-143-3p expression and the overall survival of ESCC patients. Results are expressed as the mean ± SD of three independent experiments. *: *P* <0.05; **: *P* <0.01

### Correlations between miR-143-3p expression and clinicopathological characteristics of ESCC

We next addressed the clinical significance of miR-143-3p downregulation in ESCC by evaluating correlations between miR-143-3p expression level and clinicopathological features in the 80 patients examined. Downregulation of miR-143-3p significantly correlated with advanced clinical stage and lymph node metastasis, while no significant correlations were observed for other clinicopathological parameters (Table 2). Additionally, patients with low levels of miR-143-3p expression had a poorer overall survival than those with high miR-143-3p expression (Fig. 1c). We then evaluated whether miR-143-3p could serve as an independent prognostic factor by performing univariate and multivariate analyses by the Cox proportional hazards model. Table 3 shows that miR143-3p expression level, clinical stage, and tumor differentiation all function as independent prognostic factors for these ESCC patients. Taken together, these results suggest that the downregulation of miR-143-3p may play an important role in the development and progression of ESCC.

**Table 2:** Correlation between miR-143-3p expression and clinicopathological features

Patient characteristics		MiR-143-3p expression		X^2^	*P* value
		Low (*n* = 54)	High (*n* = 26)		
Age				0.887	0.346
Median	60				
Range	38–74				
< 60	34	21(38.9 %)	13(50 %)		
≥ 60	46	33(61.1 %)	13(50 %)		
Gender				3.242	0.072
Female	18	9(16.7 %)	9(34.6 %)		
Male	62	45(83.3 %)	17(65.4 %)		
Tumor location				0.608	0.738
Upper	12	7(13 %)	5(19.2 %)		
Middle	34	23(42.6 %)	11(42.3 %)		
Lower	34	24(44.4 %)	10(38.5 %)		
Histological grade				0.547	0.761
Poor	33	22(40.7 %)	11(42.3 %)		
Moderate	31	20(37.0 %)	11(42.3 %)		
Well	16	12(22.2 %)	4(15.4 %)		
pT status				1.6222	0.444
pT1	12	10(18.5 %)	2(7.7 %)		
pT2	25	16(29.6 %)	9(34.6 %)		
pT3	43	28(20.2 %)	15(57.5 %)		
Lymph node metastasis				4.297	0.038*
Absent (0)	33	18(33.3 %)	15(57.5 %)		
Present (1/2/3)	47	36(66.7 %)	11(42.3 %)		
TNM stage				4.941	0.026*
I/II	38	21(38.9 %)	17(65.4 %)		
III	42	33(61.1 %)	9(34.6 %)		

* *p* <0.05

**Table 3:** Univariate analysis and multivariate analysis for prognostic factors in ESCC patients

Variables	Univariate analysis	Multivariate analysis		
	*P* value	HR	95 % CI	*P* value
Age (<60/≥60)	0.346	-	-	-
Gender (Female/Male)	0.22	-	-	0.785
Tumor location (Upper/Middle/Lower)	0.315	-	-	-
Clinical stage (I + II/III)	<0.001*	2.378	1.061–5.330	0.035*
Histological grade (Well/moderate/Poor)	0.045*	0.521	0.344–0.788	0.02*
Lymph node metastasis (Present/Absent)	<0.001*	1.96	0.845–4.547	0.117
MiR-143-3p expression (Low/High)	<0.001*	0.367	0.171–0.786	0.01*

*HR* hazard ratio; *95 % CI* 95 % confidence interval, *p < 0.05

### MiR-143-3p inhibits proliferation, migration, and invasion in ESCC cells

We explored the potential biological function of miR-143-3p in ESCC by stably-transfecting miR-143-3p and anti-miR-143-3p expression constructs in ESCC cell lines. Successful expression of miR-143-3p in stable transfectants was confirmed by real time RT-PCR (Fig. 2a). Overexpression of miR-143-3p decreased ESCC cells proliferation, as shown by MTT assays (Fig. 2b) and colony formation (Fig. 2c). Conversely, downregulation of miR-143-3p promoted colony-formation efficiency and cell survival (Fig. 2b, and d). Additionally, overexpression of miR-143-3p resulted in a significant increase in Annexin-V positive cells, whereas inhibition of miR-143-3p expression reduced apoptosis (Fig. 2e–f).

**Fig. 2:** MiR-143-3p has a strong tumor suppressive effect on ESCC cells growth in vitro. **a** Real time RT-PCR analysis of the relative expression of miR-143-3p in each group of stably-transfected ESCC cells. **b**–**d** Colony formation and MTT assays in ESCC cells overexpressing or underexpressing miR-143-3p. **e**–**f** Flow cytometric analysis of Annexin V-FITC staining was used to quantify apoptosis induced by miR-143-3p. Results are expressed as the mean ± SD of three independent experiments. *: *P* <0.05;**: *P* <0.01

We next investigated the influence of miR-143-3p on tumor invasion and metastasis. The wound healing assay demonstrated that the migratory ability of ESCC cells stably transfected with miR-143-3p was significantly lower than that of cells transfected with miR-NC (Fig. 3a). We then investigated whether cell mobility suppression was simply the product of an inhibitory effect on tumor cell growth, by performing an invasion assay finding that miR-143-3p suppressed the invasive ability of ESCC cells. Similarly, cell invasion was reduced in miR-143-3p-transfected cells as determined by the matrigel invasion assay (Fig. 3b). These results indicate that miR-143-3p could effectively suppress the growth, migration and invasion of ESCC cells in vitro.

**Fig. 3:** MiR-143-3p suppresses the migration and invasion of ESCC cells in vitro. **a** Wound-healing assay showed that ectopic expression of miR-143-3p effectively suppressed cell motility. **b** Migration assay and Invasion assay revealed that the ectopic expression of miR-143-3p inhibited the invasion ability of ESCC cells. Results are expressed as the mean ± SD of three independent experiments. *: *P* <0.05; **: *P* <0.01

### QKI is a potential target of miR-143-3p

We next investigated the mechanisms by which miR-143-3p inhibits ESCC cell proliferation, migration, and invasion, and five genes were selected as potential targets of miR-143-3p based on analyses of publicly-available databases. Among these genes, QKI exhibited obviously upregulaed in ESCC cell lines (Additional file 1: Figure S1). Moreover, we used a dual-luciferase reporter system to demonstrate that miR-143-3p binds directly to the 3’-UTR of QKI (Fig. 4a). Co-transfection with miR-143-3p-expressing vector significantly inhibited luciferase activity driven by the reporter vector containing the wild-type QKI 3’-UTR but not the mutant 3’-UTR. Furthermore, overexpression of miR-143-3p decreased QKI protein levels in ESCC cells, while downregulation of endogenous miR-143-3p increased QKI protein expression (Fig. 4b). These results demonstrate that miR-143-3p suppressed the expression of QKI in ESCC by directly targeting the QKI 3’-UTR.

**Fig. 4:** MiR-143-3p negatively regulates the expression of QKI by directly targeting the QKI 3’-UTR. **a** Luciferase activity in cells following co-transfection with control or miR-143-3p-encoding plasmids and wild-type or mutant-type pMIR vectors harboring the predictive miR-143-3p binding site in the 3’-UTR of QKI. **b** Western blot analysis showed that miR-143-3p could inhibit the protein expression of ESCC cells. **c** Real time RT-PCR analysis of QKI expression in human ESCC tissue samples and their matched normal tissues from ESCC patients (*n* = 80). Expression levels are shown using a log_2_ scale. **d** RT-PCR analysis of QKI mRNA expression in ESCC cells compared with that in the normal esophageal epithelial cell line (HEEC). **e** Immunohistochemical staining of QKI protein in primary ESCC tissue samples (Left: ×100; Right: ×200). **f** Analysis of correlation between QKI and miR-143-3p expression levels in 80 pairs of ESCC tissue specimens. **g** RT-PCR analysis of the expression of the major QKI splice variants regulated by miR-143-3p. Values are mean ± SD; *: *P* <0.05; **: *P* <0.01

The association between miR-143-3p and QKI was further investigated by measuring levels of QKI mRNA and protein in the primary ESCC samples and also the cell lines using real time RT-PCR and immunohistochemical staining. Figure 4c–d reveals that the expression levels of QKI mRNA were significantly higher in ESCC tumor tissues and cells compared with normal tissue and control cells, respectively. And among 80 ESCC samples, 62 were positive for QKI protein and 18 were negative. It is noteworthy that the expression levels of QKI protein were significantly higher in tumor tissues than in matched adjacent normal tissues (Fig. 4e). Furthermore, the inverse association between miR-143-3p and QKI was significant based on linear regression analysis (Fig. 4f).

We next investigated which of the QKI splice variants is important for miR-143-3p-mediated tumor-suppression by further analyzing the mRNA expression levels of QKI-5, QKI-6, and QKI-7 in cells. Overexpression of miR-143-3p markedly downregulated QKI-5 mRNA expression, whereas miR-143-3p downregulation increased QKI-5 mRNA expression (Fig. 4g). Collectively, these results suggest that the tumor suppressive effect of miR-143-3p occurred via suppression of QKI-5 expression.

### Effects of QKI-5 on ESCC cell proliferation, colony formation, migration, and invasion in vitro

We next performed functional studies using cells stably transfected with pLenti QKI-5 and pLenti siQKI-5 to stably overexpress or deplete QKI-5, respectively. QKI-5 upregulation significantly promoted ESCC cell viability and colony formation (Fig. 5a and b), while silencing of QKI-5 expression suppressed cell growth (Fig. 5b and c). Additionally, downregulation of QKI-5 significantly increased apoptosis compared with the control group (Fig. 5d).

**Fig. 5:** Knockdown of QKI-5 inhibits ESCC cell growth and induces cell apoptosis. **a**, **b** Overexpression of QKI-5 led to stronger colony formation ability and cell growth rate. **b**, **c** Downregulation of QKI-5 suppressed ESCC cell colony formation and proliferation ability. **d** Flow cytometric analyses of Annexin V-FITC staining were used to quantify apoptosis rate induced by QKI-5. Values are the mean ± SD; *: *P* <0.05;**: *P* <0.01

We next determined whether QKI-5 could affect the migration and invasion of ESCC cells. Wound healing assay showed that downregulation of QKI-5 inhibited the migratory activity of ESCC cells (Fig. 6a). Meanwhile, Invasion assay demonstrated that inhibition of QKI-5 expression reduced the invasiveness of ESCC cells (Fig. 6b). Consistently, matrigel invasion assay identified a significant reduction in cell invasion by pLenti siQKI-5-transfected cells compared with control cells (Fig. 6b). Taken together, these observations demonstrate that QKI-5 can promote ESCC progression by enhancing cell proliferation, invasion, and migration.

**Fig. 6:** Knockdown of QKI-5 inhibits ESCC cell growth and motility in vitro. **a** Wound healing assays were used to evaluate the motility of ESCC cells transfected with pLenti siQKI-5. **b** Migration assay and invasion assay were conducted in ESCC cells transfected with pLenti siQKI-5. Values are the mean ± SD; *: *P* <0.05; **: *P* <0.01

### QKI-5 is involved in miR-143-3p-mediated regulation of ESCC cell growth, apoptosis, migration, and invasion

We next investigated the mechanism underlying the tumor suppressive effect of miR-143-3p and evaluated whether QKI-5 is involved in this process by stably co-transfecting Kyse70 and Eca109 cells with miR-143-3p-expressing and pLenti QKI-5 constructs with full length QKI-5 or relevant control. MTT and colony formation assays showed that miR-143-3p overexpression decreased both cell growth rate and colony formation ability, whereas co-transfection of miR-143-3p and pLenti QKI-5 significantly blocked this anti-growth effect (Fig. 7a and b). Consistently, Fig. 7c reveals that apoptosis was significantly increased in cells transfected with miR-143-3p or miR-143-3p/pLenti-Blank compared with pLenti QKI-5-transfected cells. Furthermore, migration and invasion analyses demonstrated that cells co-transfected with miR-143-3p and pLenti QKI-5 had increased migratory and invasive capacities compared with cells transfected with miR-143-3p (Fig. 7d and e). These findings demonstrate that QKI-5 is a functional target of miR-143-3p and that ectopic expression of QKI-5 can reverse the anti-tumor effect of miR-143-3p.

**Fig. 7:** Restoration of QKI-5 reverses miR-143-3p-mediated inhibition of ESCC cell growth and metastasis. **a**, **b** MTT and colony formation assays were conducted to evaluate the proliferative capacity of ESCC cells. **c** Flow cytometric analysis of Annexin V-FITC staining was used to quantify apoptosis rate in miR-143-3p and miR-143-3p/pLenti QKI-5 group cells. **d** Migration and invasion assay were conducted in ESCC cells transfected with miR-143-3p or co-transfected with pLenti QKI-5. **e** Wound healing assays were used to evaluate the motility of ESCC cells transfected with miR-143-3p alone or co-transfected with pLenti QKI-5. Results are expressed as the mean ± SD of three independent experiments. *: *P* <0.05;**: *P* <0.01

### MiR-143-3p regulates tumor growth and apoptosis via suppression of QKI-5 in vivo

We investigated the role of miR-143-3p in tumor growth in vivo by subcutaneous injection of Kyse70 cells transfected as described above into the flank of nude mice. Figure 8a reveals that miR-143-3p overexpression significantly reduced the growth rate, volume, and average weight of Kyse70-derived tumors in mice. Furthermore, histological analysis of tumor sections and found that miR-143-3p-overexpressing cells exhibited increased apoptosis compared with miR-NC cells. We further examined the role of QKI-5 in tumor growth using xenograft mouse models and found that downregulation of QKI-5 attenuated the tumor growth rate and reduced tumor volume in vivo. Additionally, restoration of QKI-5 promoted proliferation and significantly increased tumor volume. Consistently, reduction of QKI-5 expression led to increased apoptosis, whereas induction of QKI-5 obviously decreased apoptosis (Fig. 8b).

**Fig. 8:** MiR-143-3p inhibits ESCC cells growth by inhibiting QKI-5 in vivo. **a** Effects of miR-143-3p on tumor growth in nude mice. Growth curves and weights of tumors resulted from injection of Kyse70 cells stably expressing with miR-143-3p in nude mice. Apoptosis was evaluated by performing a TUNEL assay using sections of the transplanted tumors (×200). **b** Effect of QKI-5 on tumor growth in nude mice. Xenograft assay with Kyse70 stable cells revealed that inhibition of QKI-5 decreased the volume of the xenograft tumors, while restoration of QKI-5 showed a proliferative tendency with significantly greater tumor volume. **c** Restoration of QKI-5 significantly reversed the suppression of tumor growth and apoptosis induced by miR-143-3p. *: *P* <0.05; **: *P* <0.01

Furthermore, Fig. 8c shows that restoration of QKI-5 expression significantly reversed the suppression of tumor growth induced by miR-143-3p. TUNEL analyses also revealed that attenuation of apoptosis enforced the expression of miR-143-3p and QKI-5. These observations clearly show that downregulation of miR-143-3p plays an important role in ESCC growth in vivo by targeting QKI-5.

### MiR-143-3p/QKI-5 interaction regulates EMT in ESCC cells

EMT has received much attention concerning its role in regulating invasion and metastasis in many cancers, including ESCC. During EMT, epithelial cells lose expression of epithelial markers and acquire a mesenchymal phenotype, resulting in enhanced invasion and metastasis [19]. We detected the protein levels of EMT markers in paired transfected cells to identify whether ESCC cells exhibit EMT molecular marker changes. Figure 9a and b demonstrate that both miR-143-3p overexpression and QKI-5 silening resulted in increased E-cadherin and β-catenin protein levels and decreased of vimentin and N-cadherin protein levels. Subsequently, we investigated EMT-related protein expression after co-transfection to explore whether QKI-5 cooperates with miR-143-3p to modulate EMT. Notably, rescue experiments demonstrated that miR-143-3p-dependent upregulation of epithelial protein markers upregulation and downregulation of mesenchymal protein markers was largely negated by overexpression of QKI-5 (Fig. 9c). Furthermore, we measured expression levels of EMT proteins in ESCC cells in vivo using immunohistochemistry analysis resected tumor tissue sections. Consistently, staining of E-cadherin and β-catenin protein was greatly increased in the miR-143-3p and pLenti siQKI-5 transfected groups, whereas vimentin and N-cadherin protein staining was diminished (Fig. 10a). These studies show that both miR-143-3p induction and QKI-5 suppression consistently led to stabilization of the epithelial phenotype of ESCC cells. Similarly, E-cadherin and β-catenin protein levels in the pLenti QKI-5 group were decreased compared with the miR-143-3p group (Fig. 10b). These results support a role for miR-143-3p/QKI-5 axis in modulating EMT processing in ESCC progression.

**Fig. 9:** MiR-143-3p/QKI-5 interaction regulates EMT in ESCC cells. **a**, **b** Western blotting analysis of the protein levels of EMT markers in ESCC cells after transfection with miR-143-3p or pLenti siQKI-5. **c**: Restoration of QKI-5 significantly reversed the suppression of EMT transition induced by miR-143-3p

**Fig. 10:** Immunohistochemistry analysis EMT markers expression in resected tumor tissue sections (×200). **a**: IHC analysis of the protein levels of EMT markers in ESCC cells after transfection with miR-143-3p or pLenti siQKI-5 in mice. **b**: Restoration of QKI-5 significantly reversed the suppression of EMT transition induced by miR-143-3p in mice

## Discussion

MiRNAs are important post-transcriptional regulators of gene expression and are involved in multiple biological processes, including tumorigenesis and metastasis. Although miRNA functions not fully understood, miRNA dysregulation plays a critical role in the initiation and progression of multiple human cancers, by acting as either oncogenes or tumor suppressors. In this study, we evaluated the relationship between miR-143-3p expression levels and the clinicopathological features and outcomes of ESCC patients. We report for the first time that miR-143-3p acts as a tumor suppressor in the development of ESCC by directly downregulating of QKI-5 expression and inhibiting EMT in cancer cells. Our findings indicate that miR-143-3p is potential therapy for ESCC.

Previous studies have reported a tumor suppressor role for miR-143 in several cancers. For example, miR-143-3p is downregulated in bladder cancer and inhibits cell growth through targeting oncogene KAS, but not ERK-5 [20]. MiR-143 is also downregulated in cervical cancer, enabling promotion of apoptosis and inhibition of tumor formation through targeting of Bcl-2 [21]. Furthermore, a recent report demonstrated that miR-143-5p, another member of the miR-143 family, directly targets COX-2 in gastric cancer to promote a greater growth inhibitory effect and a higher apoptotic rate than miR-143-3p [22]. Consistently, we found miR-143-3p to be aberrantly downregulated in ESCC. Ectopic expression of miR-143-3p significantly suppressed ESCC cells proliferation, induced apoptosis, and inhibited growth of xenograft tumors in nude mice, indicating that miR-143-3p acts as a tumor suppressor in ESCC. Furthermore, our research also reveals that enforced expression of miR-143-3p effectively represses cells migratory and invasive abilities.

We investigated the mechanisms underlying in miR-143-3p induced inhibition of ESCC proliferation and metastasis by conducting in silico analysis and dual-luciferase reporter assay and identified QKI-5 as a direct downstream target gene of miR-143-3p. QKI is a member of the signal transduction and activation of RNA (STAR) family, and affects pre-mRNA splicing [23], mRNA turnover [24] and translation [25]. QKI is implicated in diseases including ataxia, schizophrenia, inflammation, and multiple cancers [26–29]. Additionally, QKI is associated with tumor initiation and progression, acting as a tumor suppressor gene under the direct control of p53 in glioblastoma multiforme [30]. Levels of QKI expression are significantly decreased in some cancer tissues. For example, QKI expression correlates well with the clinicopathologic characteristics and prognosis of gastric cancer, with reduced proliferation of GC cells in vitro associated with overexpression of QKI [31]. Furthermore, QKI-5 isoform has also been identified as a tumor suppressor in oral squamous cell carcinoma [32], prostate cancer [16] and lung cancer [33]. Contrasting with these observations in other cancer types, our data demonstrate dramatic upregulattion of QKI in ESCC tissues and cell lines, and a correlation between QKI expression levels and tumor metastasis and prognosis in ESCC patients. Disrupting QKI expression, especially the QKI-5 isoform, also inhibited ESCC cells proliferation and induced cell apoptosis in vitro. Furthermore, the inhibitory effects of miR-143-3p on ESCC cell proliferation, migration, and invasion were reversed by restoration of QKI-5 expression, demonstrating the important contribution of QKI-5 in responses triggered by miR-143-3p.

Gene dysregulation plays a critical role in the initiation and progression of multiple human cancers. And many genes are identified to have dual roles as either oncogenes or tumor suppressors in different cancers. For example, hyperactive STAT3 is thought to be oncogenic in many cancers, and targeting IL-6/STAT3 is now a therapy for cancer treatment. However, a recent study revealed that STAT3 regulated ARF expression and suppressed prostate cancer metastasis. Similarly, although QKI-5 was characterized as a tumor suppressor in several cancers, its role in ESCC has not been clarified. According to our results we consider that QKI-5 may exert an oncogenic function in ESCC. We think our findings challenge the current discussion of the role of QKI-5 in tumor progression, further explorations will be made on the mechanisms and pathways of QKI-5 in ESCC progression.

We also assessed the expression levels of EMT regulatory proteins in ESCC cells because many cancers arise from epithelial cells and need to undergo EMT to become invasive and metastasize. Notably, levels of N-cadherin and vimentin were dramatically decreased in miR-143-3p and pLenti siQKI-5 transfected cells. Meanwhile, levels of the epithelial markers E-cadherin and β-catenin were increased in both groups of transfected cells. Consistently, the suppressive effect of miR-143-3p on EMT regulatory proteins could be rescued by co-transfection with pLenti QKI-5. Thus, the tumor suppressive role of miR-143-3p may regulate the EMT pathway in ESCC.

Our research reveals that miR-143-3p expression is downregulated in ESCC tissues and cells and inversely correlates with clinical TNM stage and lymph node metastatic status. Additionally, our in vivo and in vitro experiments demonstrate that enforced expression of miR-143-3p induces apoptosis, and suppresses cell proliferation, migration, and invasion capabilities by targeting QKI-5 in ESCC cells. Our results identify a novel tumor suppressive mechanism in ESCC, indicating that miR-143-3p may serve as a new diagnostic and prognostic biomarker for ESCC patients. Further studies in ESCC are required to more coherently define the role of this miR-143-3p-mediated molecular pathway in regulating ESCC initiation and progression.

## Conclusions

This study demonstrates that miR-143-3p exhibits a strong tumor-suppressive effect by inhibiting the expression of QKI-5. Furthermore, dysregulation of miR-143-3p is a molecular mechanisms involved in the development and progression of ESCC.

## Abbreviations

3’-UTR: 3’-untranslated regions; EA: esophageal adenocarcinoma; ESCC: esophageal squamous cell carcinoma; GAPDH: glyceraldehyde-3-phosphate dehydrogenase; IHC: immunohistochemistry; PBS: phosphate-buffered saline; RT-PCR: reverse transcription-polymerase chain reaction

## Additional file

Additional file 1: Figure S1. The relative expressions of five candidate genes of miR-143-3p in ESCC cell line.QKI is one of the most upregulated candidate genes of miR-143-3p in ESCC cell lines. Real time RT-PCR analysis of five candidate genes in three human ESCC cell lines and the normal esophageal epithelial cell line (HEEC). (TIF 42 kb)
